# Accurate Adiabatic and Diabatic Potential Energy Surfaces for the Reaction of He + H_2_

**DOI:** 10.1155/2022/7552881

**Published:** 2022-06-16

**Authors:** Jing Cao, Nan Gao, Yuxuan Bai, Dequan Wang, Ming Wang, Shaokang Shi, Xinyu Yang, Xuri Huang

**Affiliations:** ^1^Laboratory of Theoretical and Computational Chemistry, Institute of Theoretical Chemistry, College of Chemistry, Jilin University, Changchun, China; ^2^Department of Thoracic Surgery, China-Japan Union Hospital of Jilin University, Changchun, China; ^3^College of Life Science, Sichuan Agricultural University, Ya'an, China

## Abstract

The accurate adiabatic and diabatic potential energy surfaces, which are for the two lowest states of He + H_2_, are presented in this study. The Molpro 2012 software package is used, and the large basis sets (aug-cc-pV5Z) are selected. The high-level MCSCF/MRCI method is employed to calculate the adiabatic potential energy points of the title reaction system. The triatomic reaction system is described by Jacobi coordinates, and the adiabatic potential energy surfaces are fitted accurately using the B-spline method. The equilibrium structures and electronic energies for the H_2_ are provided, and the corresponding different levels of vibrational energies of the ground state are deduced. To better express the diabatic process of the whole reaction, avoid crossing points being calculated and conical intersection also being optimized. Meanwhile, the diabatic potential energy surfaces of the reaction process are constructed. This study will be helpful for the analysis of histopathology and for the study in biological and medical mechanisms.

## 1. Introduction

Helium and hydrogen atoms were the most abundant substances in the universe [1]. The heating led to the rotation and vibration of the H_2_ molecule in the universe when helium collided with H_2_ in the molecular cloud. In the interstellar medium, the formation of stars was quite closely linked to their interactions, which suggested that the interactions between helium and hydrogen atoms were of particular interesting. Therefore, the reaction between He and H_2_ was necessary to know the star formation in physics and chemistry, which was essential to understand the properties of many astrophysical objects. In addition, many researchers had constructed diabatic potential energy surfaces [2–16], so the construction of the global potential energy surfaces was an essential prerequisite for the title reaction. Which was an essential prerequisite for the study of molecular reaction kinetics.

Many years ago, the He + H_2_ reaction system was studied by experimental [17–21] and theoretical [1, 22–35] researchers. In 1963, Roberts [36] obtained the interaction energy of the HeH_2_ system at a relatively large center of charge separation. Subsequently, the interaction potential between He and H_2_ was studied by Krauss and Mies [23], who got conclusion that the forces are comparable for collisions along the centerline and along the molecular parallels. Henry and co-works [37] constructed and calculated each atom in the HeH_2_ system separately using Gaussian basis functions. The calculated 416 configurations were used to predict the van der Waals interaction between the lowest state of the helium atom and the hydrogen molecule. At the same time, Gengenbach and Hahn [20] constructed the earliest empirical potential energy surface for He-H_2_. Wilson's work [26] proposed a universal expression for the HeH_2_ potential energy surfaces with a straightforward function. Soon after that, Dove and Raynor [38] improved and optimized these potential energy surfaces. Meanwhile, they studied the collisional dissociation of He to H_2_. The ground and excited state potential energy surfaces were constructed for the HeH_2_ system by Stavros [36], who used the *ab initio* MRD CI calculation method. Up to 2003, Arnold and Peter [1] employed the *ab initio* method and calculated 20203 energy points in the interaction region of HeH_2_, which had an improvement and enhancement compared with previous scholars. Cavity-enhanced spectra of He-H_2_ were discussed by Słowiński et al. [39], and the results also showed that *ab initio* calculations could provide reference data for atmospheric spectroscopy studies. In the laboratory, the collision of hydrogen molecular and helium atoms would create ultracold molecules. Hence, the interaction between He and H_2_ was also an essential factor in determining the properties of hydrogen clusters within helium.

In order to getting the precisely potential energy surfaces, the large range is used to scan. the large basis sets (aug-cc-pV5Z) were selected, and the three energy states of the He + H_2_ system were calculated, using high-level MCSCF/MRCI. Secondly, the energy points were fitted using the B-spline method. Finally, as electrons would transfer near the interaction area, the conical intersection was optimized, and the avoided crossing points were studied. Meanwhile, the adiabatic and diabatic potential energy surfaces were constructed for this reaction system.

The study was organized as follows: in the next section, a brief overview of the theoretical calculation method; the adiabatic and diabatic potential energy surfaces of He + H_2_ were presented in the third chapter. And the simple summary and the conclusion would be shown in the fourth chapter.

## 2. Computational Methods

### 2.1. Ab Initio Calculations

The MOLPRO 2012 [40] package was used to perform all *ab initio* single-point energies at the high-level method (MCSCF/MRCI) with large basis sets (aug-cc-pV5Z) [41]. The three lowest state adiabatic potential energies were calculated in the He + H_2_ reaction system. There were 4 electrons in the orbital, including 15 active orbitals and 229 external orbitals (141A′+88A^″^). The Jacobi (*r*, *R*, *θ*) coordinates were selected for this triatomic system, which was widely used in our former studies [42–49]. The configuration coordinates (Figure 1) were illustrated to describe the reaction of the triatomic molecules.

The angle was determined from 0° to 90° with the grids at 10° for the reactants and field, and 12960 adiabatic potential energy points were calculated independently for each electronic state energy. For the products region, 21888 points were scanned at an angle of 0° to 180°. For each electronic state energy in the reactants and products, 34848 adiabatic potential energy points were measured, which guaranteed that the adiabatic potential energy surfaces were reliable. Tables 1 and 2 indicate the scan ranges of reactants and products, respectively. The B-spline method was used to fit the potential energy surface for this process. This method may be useful for the analysis of histopathology and for the study in biological and medical mechanisms.

### 2.2. Mixing Angle (*α*) Calculation

The wave functions of the three lowest states were *ψ*_1_^*a*^, *ψ*_2_^*a*^, and *ψ*_3_^*a*^respectively, and the adiabatic wave functions for the two lowest states were expressed as:

(1) $$\begin{array}{c} \left(\begin{array}{c} \Psi_{1}^{d}\\ \Psi_{2}^{d} \end{array}\right)=\left(\begin{array}{cc} \cos a & \sin a\\ -\sin a & \cos a \end{array}\right)\left(\begin{array}{c} \varphi_{1}^{a}\\ \varphi_{2}^{a} \end{array}\right), \end{array}$$

where *α* was denoted as the mixing angles, and the energy of the diabatic potential energy (*H*_*ii*_^*d*^) was obtained by fitting the adiabatic potential energy (*E*_*i*_^*a*^):

(2) $$\begin{array}{c} H_{11}^{d}=\cos^{2}{aE}_{1}^{a}+\sin^{2}{aE}_{2}^{a}, \end{array}$$

(3) $$\begin{array}{c} H_{22}^{d}=\sin^{2}{aE}_{1}^{a}+\cos^{2}{aE}_{2}^{a}, \end{array}$$

(4) $$\begin{array}{c} H_{12}^{d}=H_{21}^{d}=\sin a\cos a\left(E_{2}^{a}-E_{1}^{a}\right), \end{array}$$

(5) $$\begin{array}{c} H_{12}^{d}=H_{21}^{d}. \end{array}$$

*H*_11_^*d*^ and *H*_21_^*d*^ were the coupling energy between the two states. The ${\hat{P}}_{z}$ was the *Z* component of the dipole moment operator. The following equation was obtained:

(6) $$\begin{array}{c} \langle \Psi_{3}^{a}|{\hat{P}}_{z}|\Psi_{1}^{a}\rangle =\sin a\langle \Psi_{3}^{a}|{\hat{P}}_{z}|\varphi_{2}^{d}\rangle +\cos a\langle \Psi_{3}^{a}|{\hat{P}}_{z}|\varphi_{1}^{d}\rangle , \end{array}$$

(7) $$\begin{array}{c} \langle \Psi_{3}^{a}|{\hat{P}}_{z}|\Psi_{2}^{a}\rangle =-\sin a\langle \Psi_{3}^{a}|{\hat{P}}_{z}|\varphi_{1}^{d}\rangle +\cos a\langle \Psi_{3}^{a}|{\hat{P}}_{z}|\varphi_{2}^{d}\rangle . \end{array}$$

$\langle \Psi_{3}^{a}|{\hat{P}}_{z}|\varphi_{1}^{d}\rangle$ and $\langle \Psi_{3}^{a}|{\hat{P}}_{z}|\varphi_{2}^{d}\rangle$ were both highly symmetric matrices:

(8) $$\begin{array}{c} \langle \Psi_{3}^{a}|{\hat{P}}_{z}|\varphi_{1}^{a}\rangle =0, \end{array}$$

(9) $$\begin{array}{c} \langle \Psi_{3}^{a}|{\hat{P}}_{z}|\varphi_{2}^{a}\rangle =1. \end{array}$$

Thus, the mixing angles were obtained as:

(10) $$\begin{array}{c} a=\arctan\left(\left|\frac{\Psi_{3}^{a}\left|{\hat{P}}_{z}\right|\Psi_{1}^{a}}{\Psi_{3}^{a}\left|{\hat{P}}_{z}\right|\Psi_{2}^{a}}\right|\right). \end{array}$$

The main idea of the method for the mixing angle calculating can be used for histopathology after optimizing.

## 3. Results and Discussion

The lowest ground state and the first excited state potential energy surfaces were constructed in this reaction system with angles (including 0°, 30°, 50°, 60°, and 90°), sequentially. To more clearly and specifically display the potential energy surfaces, the lowest state energy of the He + H_2_ was shifted at 0.00 eV, and the results were analyzed as follows.

### 3.1. One-Dimensional Diatomic Adiabatic Potential Surface

Figure 2 shows the equilibrium bond length (*R*_*e*_) of the H_2_ molecule was 0.742 Å, and the dissociation energy (*D*_*e*_) was 37940.0582 cm^−1^. From the image, it was clearly found that a total of 13 vibrational states in the one-dimensional potential energy surface, and the zero point energy of the diatomic molecule was *E*(0,0) =2213.6876 cm^−1^, and the highest vibrational energy was *E*(13,0) =37553.7832 cm^−1^.

The spectroscopic constants for H_2_ are presented in Table 3. The data were found to be in good agreement with the theoretical and experimental researchers, such as Lee, Yuan, and He, which indicated that the calculations were more specific in this study.

### 3.2. Two-Dimensional Adiabatic Potential Energy Surfaces

The lowest potential energy for the He + H_2_ reaction system at *θ* =0.0° is seen in Figure 3. All the potential energy surface curves were very smooth. The self-variable for *x*, *y*, and *z* were represented by *r* (in Å), *R* (in Å), and *E* (in eV). The contour intervals of the potential energy surface were 0.40 eV. When *r* >2.0 Å and *R* >3.0 Å, the distance between contours was relatively sparse, which implies that the energy was comparable. When 1.0 Å > *r* >0.5 Å and*R* >2.5 Å was the entrance area in the reaction. The entrance part of the reaction had no reaction barrier, the potential energy surface had no minimum geometries, and there was no stable configuration. To more intuitively reflect the lowest ground state and the first excited state potential energy surfaces, we plotted the first excited state potential energy surfaces.

Figure 4 depicts the first excited state potential energy surface at *θ* =0.0°. When the He atom collision with H_2_ along a straight line, the geometry crossing a transition state TS_1_ (Panel B) would form the M_1_ (Panel A). The M_1_ configuration was *r* =1.15 Å and *R* =1.44 Å, and the energy was 11.870 eV. The energy of the TS_1_ (Panel B) was about 12.037 eV, when the distance was *R* =1.85 Å, *r* =1.06. It indicated that when He attacked with H_2_, it possibly generated a stable configuration (M_1_). Similarly, the complex (M_1_) overcame the TS_2_ (Panel C) which would form the M_2_, the complex (M_2_) with *r* =2.66 Å and *R* =2.21 Å, and the energy value was 11.610 eV. To sum up, the energy of M_2_ was 11.610 eV, which was slightly lower than the M_1_.

The character of Figure 5 exhibited the lowest state for potential energy surfaces when the angle was 30.0°. From the figure, the energy between adjacent contours was 0.40 eV in the contours plot, and the potential energy values became smaller as the value of *r* and *R* decreased. When*R* >2.5 Å and 0.5 Å < *r* <1.0 Å, which was the entrance part of the reactants. There were no obvious minimum at the lowest potential energy surface and no stable configuration in this region. In order to express this process more clearly and distinctly, we also plotted the first excited state potential energy surface. As shown in Figure 6, when *r* was in the range of 1.0 Å to 1.5 Å and *R* >3.0 Å, which was the entrance region for the reactants. As *R* gradually became smaller and *r* became larger, the potential energy surface appeared at a saddle point (TS_3_) at *r* =1.25 Å and *R* =1.73 Å, and the energy was 11.776 eV. Crossing the saddle point, a minimum (M_3_) would form gradually. The configuration of M_3_ was *r* equal to 2.65 Å and *R* equal to 0.88 Å, and the minimum energy was 10.147 eV.

When the angle was 50.0°, Figure 7 depicts the image of the potential energy surfaces of the ground state. In the region of 0.5 Å < *r* <1.0 Å and *R* >4.0 Å, which was the reaction entrance of the lowest state potential energy surface, and there was no obvious minimum and stable configuration. To better illustrate this process, we also showed the potential energy surfaces of excited state for the He + H_2_ reaction system, which was described in Figure 8. It is clear that for 1.0 Å < *r* <1.5 Å and *R* >2.5 Å, the energy hardly changes with *R*, which indicated the entrance part of the reactant. As the helium atom gradually approached the center of mass of the two hydrogen atoms, the minimum (M_4_) was formed, where at *r* =1.90 Å and *R* =0.84 Å, and the energy was 9.616 eV, which was the global minimum of the first excited state.

The lowest state potential energy surface and contour plot at *θ* =60.0° are shown in Figure 9. There was no minimum in the lowest state potential energy surface. In the range of 0.5 Å < *r* <1.0 Å and *R* >4.0 Å, the potential energy hardly changes with increasing *R*, so the region was the entrance region of the reactant. Similarly, we plotted the first excited state potential energy surface and contours plot in Figure 10. There was a complex (M_5_) formed, which had an energy value of 10.006 eV when *r* =1.77 Å and *R* =0.83 Å. It was different from the energy value of *θ* =50°. It can be seen that M_5_ was not the global minimum of the whole reaction system.

Figure 11 presents the lowest state potential energy surface of the He + H_2_ reaction system when *θ* =90.0°. It was seen that for *r* >2.0 Å and *R* >2.5 Å, there was no minimum. At the 0.5 Å < *r* <1.0 Å and at *R* >4.5 Å, which was entrance region for the reaction.  Figure 12 represents the first excited state potential energy. When the helium atom attacks the hydrogen atom along the angle of 90.0°, the entrance region was *R* >1.5 Å, 1.0 Å < *r* <1.5 Å. As the helium atoms close H_2_, they passed a transition state TS_4_, at *R* =0.65 Å and *r* =1.97 Å. Crossing this transition state, the minimum (M_6_) was formed, and it was at *r* =2.10 Å, *R* =0.46 Å. The minimum energy was 10.837 eV.

### 3.3. Two-Dimensional Diabatic Potential Energy Surfaces

#### 3.3.1. Avoid Crossing Point

As seen in Figure 13, it described the difference energy between the lowest state and the first excited state. At *r* =1.80 Å and *R* =0.77 Å, the energy interval between the two lowest states was the smallest, and the energy difference was 0.186 eV. It indicated that the diabatic reaction happens easily in this area.

#### 3.3.2. Conical Intersection Structure

The configuration of the conical intersection point was optimized and obtained with MOLPRO 2012 software, and the distance between two hydrogen atoms was 1.804 Å. The distance from the helium atom to the center of mass between the two hydrogen molecules was 0.862 Å, as shown in Figure 14.

The mixing angle formula was used to calculate the diabatic potential energies of the He + H_2_ reaction system. The kinetic characteristics of the entire reaction system were modified by the interaction zone. The adiabatic and diabatic potential energy surfaces with fixed *θ* =50.0° are shown in Figure 15. These panels (a), (b), (c), and (d) correspond to the potential energy curves, when the distance between two hydrogen atoms was equal to 1.1 Å, 1.2 Å, 1.3 Å, and 1.4 Å, respectively. When mix angle is equal to 0.0°, E_1_ = H_22_ and E_2_ = H_11_, and when the mixing angle is equal to 90.0°, adiabatic energy and diabatic energy were E_1_ = H_11_ and E_2_ = H_22_. The cross point appeared when the mixing angle was equal to 45.0°. It was seen that the *R* of the crossing point increased with *r*.

While *r* was equal to 2.20 and the angle at 50.0°, Figure 16 is the enlarged view of the conical intersection area. The path of the transition from energy H_11_ to energy H_22_ in this range was clearly visible.

#### 3.3.3. Two-Dimensional Diabatic Potential Energy Surfaces

In order to better understand the reaction process, the diabatic potential energy surfaces are expressed by Figures 17–20 for angles set as 0.0°,30.0°, 60.0°, 90.0°, respectively. The H_11_ and H_22_ represented the diabatic potential energy surfaces for the He + H_2_ reaction system at angles (including 0.0°, 30.0°, 60.0°, and 90.0°), respectively.

The diabatic potential energy surfaces in the He + H_2_ system were displayed at 0.0°, 30.0°, 60.0°, and 90.0°, where the blue part represented the H_22_ and the green part represented the H_11_. As the distance between two hydrogens (r) atoms increased, the cross point appeared, and the H_11_ of the reaction was transformed into H_22_. All the points on these crossing regions were almost located on the same straight line, which also meant that the diabatic potential energy surfaces constructed by the mixing angle formula were accurate and reliable.

The most likely reaction path for the He + H_2_ reaction system was predicted, which is illustrated in Figure 21. Firstly, the first excited helium atom attacked the ground state H_2_ molecule, which formed the intermediate with bond lengths of 1.53 Å, 1.90 Å, and 0.76 Å, respectively, and the energy was 9.62 eV. Secondly, the intermediate crossed the conical intersection, and the conical intersection bond lengths of 1.65 Å, 1.80 Å, and 0.62 Å. The configuration of conical intersection was very similar to the intermediate configuration in the first excited state for the reaction. Finally, the product is gradually produced. For this reaction, it was seen that the product of HeH (*X*^1^*Σ*_*g*_^1^)+ H was the most probable reaction path to reach the product.

## 4. Conclusion

In this paper, the potential energy points of the He + H_2_ reaction system were calculated using the MOLPRO 2012 software package, which selected the aug-cc-pV5Z basis sets, and applied the *ab initio* calculation method at the MCSCF and MRCI levels. The study calculated the region of 0°-90° for the reactants and 0°-180° for the products. A total of three lowest electronic states with 34848 potential energy points were calculated, and these energy points were fitted precisely using the B-Spline method.

First of all, based on the accurate potential energies, the diatomic potential energy curves of the H_2_ molecule were constructed. We found a total of 13 vibrational states and studied the equilibrium bond distance of H_2_ was 0.742 Å. The potential energy surface features were analyzed, which deduced that the global minimum energy of the first excited state was 9.616 eV. Meanwhile, the energy difference of two lowest states was 0.186 eV in interaction area, which was consistent with the conical intersection. Finally, the diabatic potential energy surfaces were constructed in the present work.

It was worth performing the full dynamical study with this global potential energy surface. We would continue this work in the following study [54].

## Figures and Tables

**Figure 1:** (a) Reactant Jacobi coordinate. (b) Product Jacobi coordinate.

**Figure 2:** The one-dimensional potential energy surfaces for H_2_ molecule as a function of distances r_H-H_ (in Å) and its different vibrational state energies *E*(*v*, *j*=0) (in cm^−1^).

**Figure 3:** The lowest state potential energy surface (in eV) for the reaction of He + H_2_ at *θ*=0.0° in Jacobi coordinate.

**Figure 4:** The first excited state potential energy surface (in eV) for the reaction of He + H_2_ at *θ* = 0.0° in Jacobi coordinate.

**Figure 5:** The lowest state potential energy surface (in eV) for the reaction of He + H_2_ at *θ*=30.0° in Jacobi coordinate.

**Figure 6:** The first excited state potential energy surface (in eV) for the reaction of He + H_2_ at *θ*=30.0° in Jacobi coordinate.

**Figure 7:** The lowest state potential energy surface (in eV) for the reaction of He + H_2_ at *θ*=50.0° in Jacobi coordinate.

**Figure 8:** The first excited state potential energy surface (in eV) for the reaction of He + H_2_ at *θ* = 50.0° in Jacobi coordinate.

**Figure 9:** The lowest state potential energy surface (in eV) for He + H_2_ at *θ* = 60.0° in Jacobi coordinate.

**Figure 10:** The first excited state potential energy surface (in eV) for the reaction of the He + H_2_ at *θ*=60.0° in Jacobi coordinate.

**Figure 11:** The lowest state potential energy surface (in eV) for He + H_2_ at *θ* = 90.0° in Jacobi coordinate.

**Figure 12:** The first excited state potential energy surface (in eV) for the reaction of He + H_2_ at *θ*=90.0° in Jacobi coordinate.

**Figure 13:** Avoid crossing point for the lowest state and the first excited state of He + H_2_ reaction.

**Figure 14:** The conical intersection structure for He + H_2_.

**Figure 15:** Adiabatic and diabatic potential energy surface at (a) r_H-H_=1.1 Å, (b) r_H-H_= 1.2 Å, (c) r_H-H_=1.3 Å, (d) r_H-H_=1.4 Å at *θ*= 50.0°.

**Figure 16:** Cut-out plot of the diabatic potential energy surface (in eV) as a function of distance r (in Å)

**Figure 17:** When *θ*=0.0°, diabatic potential energy surfaces (in eV) as a function of distances *r* (in Å) and *R* (in A).

**Figure 18:** When *θ*=30.0°, Diabatic petential energy surfaces (in eV) as the function of r and R (in Å) for theta=30.0° *r* (in Å) and *R* (in A).

**Figure 19:** When *θ*=60.0°, diabatic potential energy surfaces (in eV) as a function of distances *r* (in Å) and *R* (in A).

**Figure 20:** When *θ*=90.0°, diabatic potential energy surfaces (in eV) as a function of distances *r* (in Å) and *R* (in A).

**Figure 21:** The possible reaction path in the He + H_2_ reaction system.

**Table 1:** Calculation range of reactant part.

Calculation range of reactant part	
*R* (He-HH, Å)	0.4, 0.6, 0.8, 1.0, 1.1, 1.2, 1.3, 1.4, 1.5, 1.6, 1.7, 1.8, 1.9, 2.0, 2.1, 2.2, 2.3, 2.4, 2.6, 2.8, 3.0, 3.2, 3.4, 3.6, 3.8, 4.0, 4.2, 4.4, 4.6, 4.8, 5.0, 5.2, 5.4, 5.6, 5.8, 6.0
*r* (HH, Å)	0.4, 0.6, 0.7, 0.72, 0.74, 0.75, 0.76, 0.8, 1.0, 1.1, 1.2, 1.3, 1.4, 1.5, 1.6, 1.7, 1.8, 1.9, 2.0, 2.1, 2.2, 2.3, 2.4, 2.5, 2.6, 2.7, 2.8, 2.9, 3.0, 3.2, 3.4, 3.6, 3.8, 4.0
*θ* (degree)	0, 10, 20, 30, 40, 50, 60, 70, 80, 90

*R* (He-HH, Å): bond length from helium to the center of mass between two hydrogens, the unit is Å. *r* (HH, Å): bond length between two hydrogen atoms, the unit is Å.  *θ* (degree): the angle between *R* and *r*, the unit is degree.

**Table 2:** Calculation range of products part.

Calculation range of products part	
*R*′ (H-HeH, Å)	0.4, 0.6, 0.8, 1.0, 1.1, 1.2, 1.3, 1.4, 1.5, 1.6, 1.7, 1.8, 1.9, 2.0, 2.1, 2.2, 2.3, 2.4, 2.6, 2.8, 3.0, 3.2, 3.4, 3.6, 3.8, 4.0, 4.2, 4.4, 4.6, 4.8, 5.0, 5.2, 5.4, 5.6, 5.8, 6.0
*r*′ (HeH, Å)	0.4, 0.6, 0.7, 0.8, 1.0, 1.1, 1.2, 1.3, 1.4, 1.5, 1.6, 1.7, 1.8, 1.9, 2.0, 2.1, 2.2, 2.3, 2.4, 2.5, 2.6, 2.7, 2.8, 2.9, 3.0, 3.2, 3.4, 3.6, 3.8, 4.0
*θ*′ (degree)	0, 10, 20, 30, 40, 50, 60, 70, 80, 90, 100, 110, 120, 130, 140, 150, 160, 170, 180

*R*′ (H-HeH, Å): bond length from the hydrogen atom to the center of mass between helium and hydrogen, the unit is Å. *r*′ (HeH, Å): bond length between helium and hydrogen atoms, the unit is Å. *θ*′ (degree): the angle between *R*′ and *r*′, the unit is degree.

**Table 3:** Spectroscopic constants for H_2_.

*H*_2_ (*X*^1^*Σ*_*g*_^+^)	*R*_*e*_ (Å)	*D*_0_ (cm^−1^)	*D*_*e*_ (cm^−1^)
This work	0.742	35726.3706	37940.0582
Lee's work [49]	0.743	35687	37868
Yuan's work [50]	0.7414		38313.2
He's work [51]	0.7418		38186.2
Expt.	0.742 [52]	36118.06 [53]	38288 [52]

*R*_*e*_ (Å): the equilibrium bond length of the H_2_, the unit is Å. *D*_0_ (cm^−1^): the experimental dissociation energy of the H_2_, the unit is cm^−1^. *D*_*e*_ (cm^−1^): the equilibrium dissociation energy of the H_2_, the unit is cm^−1^.

## Data Availability

The authors can supply the study data.
